The article "Gear Fault Diagnosis and Life Prediction of Petroleum Drilling Equipment Based on SOM Neural Network" was published in 2022. Journal: Comput Intell Neurosci.

# Gear Fault Diagnosis and Life Prediction of Petroleum Drilling Equipment Based on SOM Neural Network

**DOI:** 10.1155/2022/9841443

**Published:** 2022-08-18

**Authors:** Linzhu Lu, Jie Liu, Xin Huang, Yongcai Fan

**Affiliations:** ^1^College of Petroleum and Chemical Engineering, Jingzhou University, Jingzhou 434000, Hubei, China; ^2^School of Chemistry and Chemical Engineering, Huanggang Normal University, Jingzhou 438000, Hubei, China; ^3^Jingzhou University, Admissions and Employment Department, Jingzhou 434000, Hubei, China

## Abstract

In order to solve the problem that variable working conditions and fault types cannot be diagnosed in gear fault diagnosis of petroleum drilling equipment, four kinds of faults, namely, gear broken tooth, gear crack, gear pitting, and gear wear, are studied in this paper. Based on the SOM neural network algorithm, an intelligent diagnosis model of gear fault is proposed, and the PCA method is used to reduce data dimension and fuse features. The state index of life prediction is determined, and the remaining service life prediction of gear transmission system is predicted based on exponential degradation model. The results show that the accuracy of the SOM model for fault diagnosis is high, and the bearing in gearbox can be replaced or repaired in advance according to the residual life curve, so as to achieve the purpose of predictive maintenance.

## 1. Introduction

With the manufacturing industry entering the “industry 4.0” era, modern mechanical equipment has absorbed the new technology of modern science and technology development, and the degree of automation of mechanical equipment has become higher. At the same time, the structure of equipment has become more complex. Therefore, higher requirements have been put forward for the safety, reliability, and maintainability of the equipment in the operation process [1, 2]. Fault diagnosis technology plays an important role in ensuring the reliability, safety, and maintainability of equipment operation.

The key transmission equipment of petroleum drilling equipment is the key part to ensure the normal operation and power transmission of the whole equipment system. However, affected by the bad working environment, heavy load, high speed, and other working conditions, some typical parts of petroleum drilling and production equipment, such as gears and rolling bearings, are prone to various types of failures, which will affect the safety and reliability of the whole petroleum drilling system. At least, it will lead to the decline of product or service quality and even cause huge economic losses and casualties. Monitor the condition of large-scale key gear transmission equipment in the petroleum industry, timely handle the faults in the operation of petroleum equipment, and ensure the safe operation of the equipment. At the same time, predicting the future operation trend and remaining service life of the equipment and carrying out equipment maintenance in advance can save maintenance costs, improve economic benefits of enterprises, avoid accidents, and ensure personnel safety [3, 4].

The article "Gear Fault Diagnosis and Life Prediction of Petroleum Drilling Equipment Based on SOM Neural Network" was published in 2022. Journal: Comput Intell Neurosci.

In the process of fault diagnosis of mechanical equipment, after obtaining equipment information, equipment fault is judged by simple time domain signal in the early stage. With the development of diagnosis technology, this simple diagnosis method cannot meet the development needs, and then more reliable and accurate modern signal processing and feature extraction methods are derived [5]. But as the amount of data storage increases, the amount of data to be processed and the corresponding feature dimension increase, these factors will make the fault database rich, but also weaken the information redundancy, data processing, and computing capacity [6]. In addition, the application of fault diagnosis in petroleum field is too few, the main research results are also mainly focused on fault diagnosis and analysis under fixed working conditions. Although the structure and principle of the petroleum gear transmission system are the same, the operation conditions of the heavy petroleum gear transmission system are complex, and there are problems of variable speed and variable load, which will increase the difficulty of fault diagnosis [7, 8]. The research on fault prediction and remaining service life prediction of petroleum drilling equipment is relatively less. Moreover, it is also found that the fault diagnosis method based on machine learning and remaining service life prediction of equipment are the development trend of petroleum drilling and production equipment [9, 10].

In order to solve the problem that variable working conditions and fault types cannot be diagnosed in the gear fault diagnosis of petroleum drilling equipment, four kinds of faults, namely, gear broken tooth, gear crack, gear pitting, and gear wear, are studied in this paper. Therefore, in view of the limitations of existing fault diagnosis methods in heavy petroleum gear fault diagnosis, this paper studies the unsupervised machine learning algorithm based on SOM for heavy petroleum gear fault diagnosis under complex working conditions.

## 2. Fault Classification of Transmission System

As the key transmission equipment of petroleum drilling and production equipment, a heavy petroleum gearbox is the key part to ensure the normal operation of the whole equipment system and transfer power. The components of gear transmission system include gears, bearings, and shafts. According to the statistics in literature [11], the gear and bearing account for 79% of failure parts. Gear failure mainly includes gear broken and crack, gear pitting, gear wear, tooth surface gluing, and tooth profile error caused by manufacturing and installation. As shown in Figure 1, this paper selects four kinds of faults: gear broken, gear crack, gear pitting, and gear wear.

The article "Gear Fault Diagnosis and Life Prediction of Petroleum Drilling Equipment Based on SOM Neural Network" was published in 2022. Journal: Comput Intell Neurosci.

### 2.1. Gear Broken

Gear broken tooth is a serious fault in gear fault. In the process of gear meshing, when the overload impact and pulse cyclic stress occur, the gear will be broken, which can be divided into two forms: overload and fatigue. The first is the tooth fracture caused by overload, which is mainly due to improper assembly. In the process of operation, the load is concentrated at one end of the gear, or the sudden stop and reversing of the gear cause impact overload, resulting in tooth fracture. The second is fatigue fracture, which is mainly caused by improper design, poor assembly, excessive or unbalanced load, stress concentration caused by surface defects of gear teeth, etc.

### 2.2. Gear Wear

Gear wear is common in gear failure. The wear is mainly divided into normal wear, medium wear, abrasive wear, interference wear, and corrosion wear. If the degree of wear does not affect the normal operation of the gear, it is generally called normal wear. Moderate wear is mainly caused by high load on the teeth. In general, the service life of the driving gear will be reduced from large to small. When the sliding of the gear meshing dividing circle is blocked, it will lead to excessive wear of the gear, which shows that the working state becomes bad, the tooth profile changes, and in serious cases, it will cause pitting corrosion and plastic deformation. When there are external particles into the gear meshing surface, it will lead to abrasive wear.

### 2.3. Gear Crack

Gear crack is an early phenomenon of gear fatigue fracture. When the petroleum film of the gear is damaged, the local stress concentration will be caused at the crack. Under the action of cyclic stress, the crack will slowly expand and eventually cause the crack to fracture. This process can be monitored and predicted where the crack appears as tearing crack on the sliding direction of the tooth surface or the appearance is a ridge shape.

### 2.4. Gear Pitting

The pitting corrosion of gears can be divided into early pitting and destructive pitting. When the surface of the gear is locally convex and bears a large load, or is affected by the high-frequency variable stress, the early pitting corrosion of the gear will be caused, which generally occurs on the surface of the tooth root near the dividing circle of the gear. When the hardness of the gear surface is low, the viscosity of lubricating petroleum is low, and when the dynamic load caused by local pitting corrosion increases, the destructive pitting corrosion of gear will be caused, which is characterized by the destruction of profile and the large size of pitting corrosion. The pitting formed by destructive pitting often becomes the fatigue source and eventually leads to the fatigue fracture of gear.

The article "Gear Fault Diagnosis and Life Prediction of Petroleum Drilling Equipment Based on SOM Neural Network" was published in 2022. Journal: Comput Intell Neurosci.

## 3. Fault Diagnosis of Transmission System based on Neural Network

### 3.1. Self-Organizing Maps (SOM) Neural Network Algorithm

SOM neural network realizes the ordered mapping from high-dimensional distribution to low-dimensional regular grid, which is often used as dimensionality reduction of data features. The output neurons of the SOM network compete with each other to be activated, so only one winning neuron is output at each time. As shown in Figure 2, in the self-organizing map, neurons are placed on the network nodes. Usually, the mesh is one-dimensional or two-dimensional, while the SOM network is different from the BP network in that it only contains input layer and competition layer. Since there is no hidden layer, the SOM network can keep the original topological structure of output layer data, which is a typical feature of the SOM network.

The formation process of SOM can be divided into four stages.

The first stage: initialization, the initial connection weights are randomly initialized and the smaller weights are selected.

The second stage of their numerical competition is called the numerical discrimination of neurons.

The third stage: cooperation, the winning neuron determines the spatial location of the topological neighborhood of the excited neuron, thus providing the basis for the cooperation of adjacent neurons.

The fourth stage: adaptation, in which the excitatory neurons increase their discriminant function value about the input pattern through the proper adjustment of their synaptic weights, and the response of the winning neurons to the later similar input patterns is enhanced. Based on the formation process of SOM, the algorithm steps of feature mapping are as follows [12]:

(1) The weight vector *W*_*j*_ is initialized randomly and the smaller weight is selected
(2) A sample *X*=(*x*_1_, *x*_2_, *x*_3_,…,*x*_*m*_)^*T*^ is randomly selected from the input space to the input layer
(3) The distance between the weight vector of each neuron and the input vector is calculated, its calculation formular is as follows:
  (1) $$\begin{array}{c} d_{j}=\left\|X-W_{j}\right\|=\sqrt{\sum_{i=1}^{m}{\left(x_{i}\left(\left(t\right)-w_{ij}\left(t\right)\right)\right)}^{2}}, \end{array}$$
  where *w*_*ij*_ is the weight between *i* neuron at the input layer and *j* neuron at the mapping layer. Through calculation, a neuron with the minimum distance is obtained, which is called the winning neuron and denoted as *j*^*∗*^, that is, a certain unit *k* is determined, such that *d*_*k*_=min_*j*_(*d*_*j*_) for any *j*. And the set of adjacent neurons is obtained.
(4) Modify the weights of output neurons and their adjacent neurons
  (2) $$\begin{array}{c} \Delta w_{ij}=w_{ij}\left(t+1\right)-w_{ij}\left(t\right)=\eta \left(t\right)\left(x_{i}\left(t\right)-w_{ij}\left(t\right)\right), \end{array}$$
  where *r* is a constant greater than 0 and less than 1, which gradually decreases to 0 as time changes.
  (3) $$\begin{array}{c} \eta \left(t\right)=\frac{1}{t}\text{or }\eta \left(t\right)=0.2\left(1-\frac{t}{10000}\right). \end{array}$$
(5) Calculate the output
  (4) $$\begin{array}{c} o_{k}=f\left(\underset{j}{\min}\left\|X-W_{j}\right\|\right), \end{array}$$

where *f*(*∗*) is generally 0∼1 function or other nonlinear functions.

The article "Gear Fault Diagnosis and Life Prediction of Petroleum Drilling Equipment Based on SOM Neural Network" was published in 2022. Journal: Comput Intell Neurosci.

### 3.2. Signal Extraction

Before the fault intelligent diagnosis of heavy petroleum gear, it is necessary to complete the feature extraction of fault vibration signal due to the fact that the internal parts of the heavy petroleum gearbox are coupled with each other under actual working conditions, and the load under variable working conditions is complex and changeable. In order to obtain more useful fault feature information, based on the time domain feature extraction of the original signal, the modulation information affecting the sideband in different faults is extracted, and the high-frequency characteristics are filtered out by Hilbert envelope spectrum method, The modulation frequency information affecting the sideband is extracted from the low frequency signal, and then the feature set is formed with the time domain index characteristics of the original vibration signal, which is used as the data sample of the subsequent intelligent fault diagnosis algorithm.

#### 3.2.1. Extraction Device

The vibration data used is from the QPZZ-II rotating machinery vibration analysis and fault diagnosis test platform [13]. The data has the characteristics of various loads and variable speed. In order to collect vibration signals, nine sensors are installed in the gearbox box, and the installation position diagram is shown in Figure 3.

In order to collect vibration signals, nine sensors are installed in the gearbox box, and the installation position diagram is shown in Figure 3, where X is the radial horizontal direction and Y is the radial vertical direction. The measurement position and type of each channel are shown in Table 1.

The article "Gear Fault Diagnosis and Life Prediction of Petroleum Drilling Equipment Based on SOM Neural Network" was published in 2022. Journal: Comput Intell Neurosci.

In the experiment, the input and output frequencies of the gearbox are 5120 Hz and 880 rpm, respectively. The sampling time of each state is 10 s. The vibration signals collected by sensors 2–9 are selected. Combined with speed and gearbox related result parameters, two-stage meshing frequency and fault characteristic frequency of each gear can be obtained, as shown in Table 2.

#### 3.2.2. Sample Extraction

Under the QPZZ-II rotating machinery vibration analysis and fault diagnosis test platform, gear normal, broken teeth, pitting corrosion, and wear data are analyzed. Gear fault features are extracted from time domain, where the state can be divided into normal, broken gear, pitting, and abrasion. Eight features are selected, namely, kurtosis, RMS, ShapeFactor, MarginFactor, peak-to-peak value, waveform factor, margin factor, and energy value under the envelope frequency signal. Four samples are selected for each fault type, and a total of 16 groups of samples are selected to form SOM adaptive network learning samples. The characteristic number of envelope spectrum signal is 8, which makes up 16×. The matrix of 8 is used as the data sample of energy algorithm, as shown in Table 3.

### 3.3. Fault Diagnosis

The SOM algorithm belongs to an unsupervised algorithm. The difference between the supervised algorithm and unsupervised algorithm is that the supervised algorithm requires input data and corresponding label, while the unsupervised algorithm does not need corresponding label of input data, so it has self-learning ability and explores the internal structure of unknown data. Combined with the SOM network algorithm, the flow chart of fault diagnosis is shown in Figure 4.

Different from the supervised algorithm, the SOM network algorithm should design the number of competition layer neurons and network topology before training, and the number of output neurons will also be the final classification results. In this paper, each input is connected to 8×. There are 64 neurons in the hexagonal grid. A two-dimensional output layer composed of 64 neurons is selected, and the index value ranges from 1 to 64. The competitive position of neurons is shown in Figure 5.

### 3.4. Result Analysis

#### 3.4.1. Results of Model Training

As shown in Figure 6, when the number of training steps is 10, the number 1 and 5 of fault causes are divided into one category; 2, 6, and 7 are divided into one category; 3, 9, and 10 are divided into one category; and 13, 14, and 15 are divided into one category. It can be seen that the SOM network can classify the samples in the case of few training steps, but this classification is not accurate enough. When the number of training steps is increased, the accuracy of classification is also increased, and the SOM network has been able to accurately classify each sample when the number of training steps is increased to 100. However, when the number of training steps continues to increase, it has no effect on the classification results. For example, when the number of steps is 200 and 500, the improvement of training steps has no effect on the accuracy of the results. On the contrary, it will increase the training time.

The article "Gear Fault Diagnosis and Life Prediction of Petroleum Drilling Equipment Based on SOM Neural Network" was published in 2022. Journal: Comput Intell Neurosci.

#### 3.4.2. Results of Sample Diagnosis

Through the comparison of different training times of the SOM model, in order to exclude the influence of too few or too many training steps on the results, the training times of the model are selected as 200, and the test set data numbered 4, 8, 12, and 16 are classified with the SOM network completed by training. The results are shown in Table 4.

Comparing the diagnosis results in Table 4 with the results of 200 training steps in Figure 6, it is found that the SOM network can diagnose the fault types corresponding to the data to be tested, and the accuracy rate reaches 75%.

## 4. Life Prediction of Equipment

### 4.1. Prediction Steps

The process steps of residual life prediction of rolling bearing based on the degradation model are as follows:

  Step 1: collect the original vibration signal of rolling bearing with sensor
  Step 2: extract and calculate the eigenvalues by using vibration signal processing and analysis technology and smooth the extracted features
  Step 3: divide the training set and take the early data of the data set as the training data
  Step 4: evaluate the features, use PCA technology to reduce the dimension of the data, and perform data fusion
  Step 5: select the status index
  Step 6: fitting the degradation model of the remaining service life of the training data to obtain the fitting degradation model
  Step 7: use the fitting degradation model to predict the residual life

### 4.2. State Index Selection

The extraction of the original vibration signal of rolling bearing is the same as before, so the selection of state index is directly described. Among the first six features with large monotonicity, only the peak-to-peak value has better monotonicity. However, if only it is selected as the state index, the information of original data will be lost and error analysis will be caused. Therefore, PCA is used to analyze and fuse multiple features extracted from original data, and the largest principal component is taken as the indicator of state. Through the PCA analysis of vibration signal, the state index is obtained as shown in Figure 7. The value of state index increases gradually with time, and it can be seen from the growth trend that the state index has a monotonic increasing trend, which can be used to fit the degradation model.

The article "Gear Fault Diagnosis and Life Prediction of Petroleum Drilling Equipment Based on SOM Neural Network" was published in 2022. Journal: Comput Intell Neurosci.

### 4.3. Prediction Results

When the state index is selected, the exponential degradation model is used to fit the residual life degradation model of bearing. The model can predict the remaining service life of bearing in real time. The exponential degradation model predicts the remaining service life according to its prior parameters and measured values:

  The parameter values are defined as follows: *E*(*θ*)=1, Var(*θ*)=10^6^, *E*(*β*)=1, Var(*β*)=10^6^.

The exponential degradation model also provides a function to evaluate the slope. Once the slope of the state index changes significantly, the model will forget the previous observation results and reestimate based on the original prior value. When the slope detection value is adjusted continuously in the model fitting, the final value is 0.025 that the model has the best effect. The degradation model obtained by fitting is shown in Figure 8.

After the model fitting is completed, the life prediction of the data is carried out, and the remaining service life of the bearing is predicted by comparing the threshold value of the input measured value with the final failure threshold value. The residual life curve is shown in Figure 9.

The actual life curve (blue) and predicted life curve (red) show that the slope of input state index changes at 37 min. Before that, the change of slope cannot be detected in this time area because the change of state index is not obvious. After 37 min, the life curve changes obviously, and the life is 0 at 51 min, reaching the failure threshold one day earlier than the actual life. According to the predicted residual service life curve, the equipment can be maintained in advance and the bearing can be replaced to prevent accidents.

## 5. Conclusion

In view of the limitations of the existing fault diagnosis methods in gear fault diagnosis of heavy petroleum drilling, this paper proposes a gear fault intelligent diagnosis model based on the SOM neural network algorithm. Under this model, the data not entered into the label are classified. 16 groups of data samples are selected and 8 characteristic indexes are selected. Experimental results show that the accuracy rate of fault classification is 75%. In addition, based on the degradation model, the remaining useful life of drilling equipment is predicted. The results show that the obvious change of slope can be detected at 37 min, which verifies the effectiveness of the exponential degradation model. The bearing in gearbox can be replaced or repaired in advance according to the residual life curve, so as to achieve the purpose of predictive maintenance.

The article "Gear Fault Diagnosis and Life Prediction of Petroleum Drilling Equipment Based on SOM Neural Network" was published in 2022. Journal: Comput Intell Neurosci.

## Figures and Tables

**Figure 1:** Fault classification of the transmission system.

**Figure 2:** SOM network structure.

**Figure 3:** Installation position of sensors.

**Figure 4:** Fault diagnosis process of the SOM network.

**Figure 5:** Location of neurons in the competitive layer.

**Figure 6:** Clustering results of the model.

**Figure 7:** Status indicators.

**Figure 8:** Degradation model.

**Figure 9:** Residual life curve of equipment.

**Table 1:** Measurement position and type of sensors.

Serial number	Channel	Type	Position
1	TACH1	Speed, photoelectric	Input shaft
2	CH1	Displacement	Input shaft *X* direction displacement
3	CH2	Displacement	*Y* direction displacement of input shaft
4	CH3	Acceleration	Input shaft motor side bearing *Y* direction
5	CH4	Acceleration	Output shaft motor side bearing *Y* direction
6	CH5	Acceleration	Input shaft load side bearing *Y* direction
7	CH6	Acceleration	Output shaft load side bearing *Y* direction
8	CH7	Acceleration	Output shaft motor side bearing *X* direction
9	CH8	Magnetoelectric acceleration	*X* direction of bearing on load side of output shaft

**Table 2:** Characteristics of gear fault.

	G1	G2
Speed (rpm)	880	880
Meshing frequency (Hz)	806	806
Gear shaft rotation frequency (Hz)	14.67	10.75
Modulus	2	2
Number of teeth	55	75

**Table 3:** Sample data of SOM algorithm.

Working condition	Number	1	2	3	4	5	6	7	8
Normal	1	4.8204	5.4538	1.3249	1.6298	22.7901	1.7988	11.9818	776444.4
	2	4.9564	3.9660	1.2248	1.5282	10.2257	4.5461	11.5586	74443.0
	3	3.3134	3.5523	1.2034	0.9806	5.0575	10.2814	15.9342	11443.0
	4	5.8960	3.7342	1.1651	1.9874	0.1924	7.3950	17.6332	17344.2

Broken gear	5	7.0881	3.8081	1.3260	3.1636	15.4171	3.5039	7.1462	154360.0
	6	4.1284	5.7812	1.2990	1.7334	21.1364	3.1244	5.1195	288630.0
	7	4.0225	3.7241	1.2631	2.1591	11.2343	3.7386	9.4664	92477.0
	8	3.8737	3.9982	1.2519	1.6157	12.1311	3.9084	9.9526	105970.0

Pitting	9	18.4485	4.2961	1.3399	6.5161	32.5243	4.7026	17.3040	161890.0
	10	13.8548	5.2683	1.4125	3.6196	28.1052	3.2914	10.1228	362930.0
	11	15.6913	4.2410	1.3865	4.7952	21.6414	3.8384	16.4008	201850.0
	12	21.7750	4.2334	1.3950	6.2305	22.8853	4.2299	21.3788	192410.0

Abrasion	13	2.6554	6814.4	1.0001	0.0001	40.2643	4710.3	17.8188	221550.0
	14	2.5848	6827.7	1.0001	0.0001	37.0109	4819.0	16.9743	208020.0
	15	2.6557	6835.2	1.0001	0.0001	32.9251	5019.1	16.2253	197220.0
	16	1.7965	6693.4	1.0001	0.0001	34.0624	5176.3	17.7266	217170.0

**Table 4:** SOM diagnosis results.

	Normal	Broken gear	Pitting	Abrasion
Serial number to be tested	1	5	9	13
Diagnosis results	59	30	8	1

The article "Gear Fault Diagnosis and Life Prediction of Petroleum Drilling Equipment Based on SOM Neural Network" was published in 2022. Journal: Comput Intell Neurosci.

## Data Availability

The dataset can be accessed upon request.
